This article has been retracted.

# Influencing Factors of Physical Activity in Patients with Lung Cancer Surgery and Its Correlation with Exercise Self-Efficacy and Perceived Social Support

**DOI:** 10.1155/2022/7572530

**Published:** 2022-07-19

**Authors:** Na Zhang, Xin He, Huanhuan Zhang, Yajing Zhu, Yan Liu

**Affiliations:** Department of Thoracic Surgery, National Cancer Center, National Clinical Research Center for Cancer, Cancer Hospital, Chinese Academy of Medical Sciences and Peking Union Medical College, Chaoyang District, Beijing 100021, China

## Abstract

**Purpose:**

The aim of the study is to understand the current status of physical activity in patients with lung cancer surgery, explore its influencing factors, and analyze the correlation between physical activity and exercise self-efficacy and perception of social support.

**Methods:**

The General Information Questionnaire was designed for 145 patients, Chinese version of EPIC-PAQ physical activity scale for lung cancer patients. The Exercise Self-Efficacy Scale (SEE) is used to evaluate the ability of people to organize and execute motor behaviors in various difficult situations. The Perceived Social Support Scale (PSSS) was used to emphasize individual self-understanding and self-feeling.

**Results:**

The median and quartile of total physical activity scores in lung cancer surgery patients were 73.0 (34.8, 129.7) points; univariate analysis showed that there were statistically significant differences in physical activity levels among lung cancer surgery patients with different ages, work status before hospitalization, and perceived disease severity. The results of multivariate analysis showed that age, perceived disease severity, exercise self-efficacy, and total score of perceived social support affected the physical activity level of patients (*P* < 0.05). Efficacy were positively correlated with perceived social support (*P* < 0.01).

**Conclusion:**

The level of physical activity of patients undergoing lung cancer surgery needs to be further improved. Physical activity is affected by patient age, perceived disease severity, exercise self-efficacy, and perceived social support and is positively correlated with exercise self-efficacy and perceived social support. Medical staff should provide targeted activity guidance according to the age and other characteristics of patients undergoing lung cancer surgery, enhance patients' exercise self-efficacy and comprehend social support, and improve their physical activity level, thereby promoting patients' early recovery.

## 1. Introduction

Lung cancer is the most common malignant tumor in the world. According to the latest data from the National Cancer Center, lung cancer is the malignant tumor with the largest number of morbidities and deaths in my country [1]. Surgery is one of the main treatments for lung cancer patients. Physical activity (PA) refers to any physical activity that results in energy expenditure due to skeletal muscle movement [2]. The American College of Sports Medicine (ACSM) and the American Cancer Society have recommended physical activity as an intervention to help cancer survivors cope with pain, improve quality of life, and potentially prolong survival [3]. Research evidence shows [4–8] that regular and appropriate physical activity has a good effect on the primary prevention of cancer patients, prolonging survival time, and improving quality of life. Physical activity can improve cardiopulmonary function, improve body composition, reduce fatigue, relieve anxiety and depression, and improve the quality of life of cancer survivors. Although physical activity has many benefits for cancer patients, studies have shown [9] that nearly 2/3 of cancer patients do not meet the recommended amount of physical activity. Strategies to increase physical activity in cancer patients include encouraging physical activity practice, changing patient self-efficacy, and encouraging social support [10, 11]. The purpose of this study is to understand the current status of physical activity, exercise self-efficacy and perception of social support in patients with lung cancer surgery, and to explore the influencing factors of physical activity and the relationship between the three, so as to provide medical staff with more targeted activities and health care for patients with lung cancer surgery. Guidance provides the basis for enhancing the patient's exercise self-efficacy and social support, improving their physical activity level, and promoting the patient's early recovery.

## 2. Materials and Methods

### 2.1. Research Subjects

Patients with lung cancer who were hospitalized in the Department of Thoracic Surgery of our hospital for surgical treatment from February to April 2022 were selected as the research subjects. Inclusion criteria were as follows: ① those who met the diagnostic criteria for lung cancer in the “Chinese Standards for the Diagnosis and Treatment of Primary Lung Cancer (2015 Edition)”, and be diagnosed by pathological examination; ② aged 18–75 years old; ③ clear consciousness, no cognitive function, and communication impairment; ④ know their condition and diagnosis; and ⑤ those who submitted informed consent and are willing to participate in this study. Exclusion criteria were as follows: ① has metastasized to other parts, affecting systemic function; ② has a severe mental disorder, language communication disorder, and cognitive impairment; and ③ voluntarily withdrawn from the researcher.

### 2.2. Methods

#### 2.2.1. Survey Tools

*(1) General Information Questionnaire*. General Information Questionnaire was designed for 145 patients including general demographic information such as age, gender, occupation, education level, and per capita monthly income of the family, and disease-related information such as disease course, lesion size, and surgical method.

*(2) Chinese version of EPIC-PAQ physical activity scale for cancer patients*. It was obtained by Shujin et al. [12] Chinese translation of the EPIC Physical Activity Questionnaire (EPIC-PAQ) developed by the European Nutrition and Cancer Prospective Cohort Research Organization. The test-retest reliability of the Chinese version of the Physical Activity Scale for Cancer Patients was 0.818, the content validity index was 0.900, and the criterion validity was 0.417. The Physical Activity Scale for Cancer Patients includes 3 dimensions and 4 questions of occupational physical activity, housework physical activity, and leisure time physical activity. There are 6 kinds of physical activities in the second question, so there are 9 items in the whole questionnaire. EPIC assigns metabolic equivalents (METs) to each physical activity. We divide the population into 4 categories based on work status and leisure time physical activity time: Insufficient physical activity-sedentary work, no recreational activities; mild insufficiency of physical activity-sedentary work with less than 0.5 hours of recreational activity per day or standing work with no recreational activity. Moderate physical activity-sedentary work with 0.5 to 1 hour of recreational activity per day or standing work with 0.5 hour of recreational activity per day or physical work with no recreational activity; physically active-sedentary work with more than 1 hour of recreational activity per day or standing work with >0.5 hours of recreational activity per day or physical work or heavy manual work with at least some recreational activity [13].

*(3) Exercise Self-Efficacy Scale (SEE)*. The SEE developed by Bandura, translated, and revised by Taiwan scholar Lee et al. [14] is used to evaluate the ability of people to organize and execute motor behaviors in various difficult situations. The scale contains 18 items, each graded on a scale of 0 to 100, with 100 representing full confidence, 50 representing half confidence, and 0 representing no confidence at all. The exercise self-efficacy score is the sum of the scores for each assessment item and then divided by the total number of items. A higher score indicates a higher level of exercise self-efficacy. The reliability of the scale is between 0.82 and 0.96.

*(4) Perceived Social Support Scale (PSSS)*. This scale is a social support scale that emphasizes individual self-understanding and self-feeling. For the degree of support from friends and others, Cronbach's alpha coefficient is 0.922, using a scale of 1 to 7, and the total score reflects the overall degree of social support felt by individuals [15].

#### 2.2.2. Survey Methods

This questionnaire is distributed when patients with lung cancer surgery are discharged from the hospital. Before distributing the questionnaires, the distribution personnel will be trained uniformly through group meetings to make them understand the content of the questionnaires. According to the inclusion and exclusion criteria, the questionnaire star QR code was issued to the lung cancer patients who met the requirements, and the patients scanned the code to fill in the questionnaire by themselves. In the process of distributing the questionnaire, it is necessary to obtain the informed consent of the patients, use a unified guide language to explain the purpose and significance of this research to the patients, fill in anonymously, and explain the filling requirements on the first page of the questionnaire. For patients who are unable to complete the questionnaire, their immediate family members will fill it out on their behalf. A time limit was set for answering questions on WeChat, and you can submit it only after filling in no missing items.

### 2.3. Statistical Analysis

SPSS 24.0 statistical software was used for statistical analysis. The enumeration data were expressed as the number of cases and the composition ratio (%). The measurement data conforming to the normal distribution are expressed as the mean ± standard deviation, the nonnormally distributed data are expressed as the median (quartile) (M (P25, P75)), and the chi-square test and rank sums are used for comparison between groups. Unordered multiclass logistic regression analysis was used to explore the main influencing factors of physical activity in patients with lung cancer surgery. The relationship between physical activity and exercise self-efficacy and perceived social support was analyzed by the Pearson correlation. *P* < 0.05 was considered to be statistically significant.

### 2.4. Ethical Review

This study has been approved by the Ethics Committee of the National Cancer Center/Peking Union Medical College Cancer Hospital, Chinese Academy of Medical Sciences (approval number: 21/018–2689).

## 3. Results

### 3.1. Physical Activity of Patients with Lung Cancer Surgery

The results showed that the total physical activity score of patients after lung cancer surgery was 9.0–310.0 points, and the median and quartile were 73.0 (34.8, 129.7) points. There were 43 cases of insufficient/mild insufficiency of physical activity, accounting for 29.7%; physical activity was moderate in 58 cases, accounting for 40.0%. Physical activity was active in 44 cases, accounting for 30.3%.

### 3.2. Scores of Exercise Self-Efficacy and Perceived Social Support in Patients with Lung Cancer Surgery

The results showed that after lung cancer surgery, the median and quartile of exercise self-efficacy were 90.0 (45.5, 155.0) points and the median and quartile of perceived social support were 64.0 (48.5, 74.5) points.

### 3.3. Univariate Analysis of Physical Activity Levels in Patients with Different Characteristics of Lung Cancer Surgery

A total of 146 questionnaires were distributed, of which 145 were collected and collated. The results showed that there were statistically significant differences in physical activity levels among lung cancer patients with different ages, work status before hospitalization, and perceived disease severity (*P* < 0.05), as shown in Table 1.

### 3.4. Unordered Multiclass Logistic Regression Analysis of Influencing Factors of Physical Activity in Patients with Lung Cancer Surgery

With physical activity level as the dependent variable, age, prehospital work status, perceived disease severity, exercise self-efficacy, and perceived social support total score as independent variables, unordered multi-category logistic regression analysis was performed. The results showed that age, perceived disease severity, exercise self-efficacy, and perceived social support total score affected the level of physical activity in patients with lung cancer surgery (*P* < 0.05). See Tables 2-3.

### 3.5. Correlation Analysis of Physical Activity Level with Sport Self-Efficacy and Understanding Social Support in Patients with Lung Cancer Surgery

The results showed that physical activity was positively correlated with exercise self-efficacy and perceived social support in patients with lung cancer surgery (*P* < 0.01), as shown in Table 4 and Figures 1–2.

## 4. Discussion

It can be seen that the exercise level of lung cancer patients is not optimistic, which is consistent with the results of many studies. The study of Williams et al. [16] showed that the physical activity of lung cancer patients is lower than that of ordinary people, and the physical activity is less after diagnosis, and more is just sitting. Feng Liyan et al. [17] surveyed 191 lung cancer patients during chemotherapy and showed that only 6.81% of the patients reached the recommended amount of exercise and 67.02% of the patients were at a low level of exercise; A longitudinal study by Lin et al. [18] showed that 36% of lung cancer patients reported reduced or stopped walking exercise in the past 6 months. The reasons for the analysis are related to many factors such as the patient's physiology, psychology, and social culture, including the patient's physical condition, living habits, psychological condition, medical staff guidance, time factors, and environmental factors [19]. Studies have shown that physical activity can produce a series of benefits for lung cancer patients, which can improve the cardiopulmonary and fatigue status of lung cancer patients, and improve the survival rate [20, 21]. We reduce physical and mental fatigue, reduce anxiety, increase cognitive function, improve self-esteem, increase muscle tone and balance, help weight control, enhance immune system, improve sleep, improve quality of life, etc. [22–24]. The American College of Sports Medicine (ACSM) recommends that cancer patients do at least 150 minutes of moderate-intensity or 75 minutes of vigorous-intensity exercise per week [25]. In view of the fact that the level of physical activity of patients undergoing lung cancer surgery needs to be improved, medical staff and patients should pay more attention to physical activity and formulate a reasonable exercise program according to the specific situation of the patient to improve the physical activity level of the patient.

Young and middle-aged patients are more likely to suffer from insufficient physical activity, and patients with less severe disease are more active in physical activity. The reasons for this analysis may be that the incidence of lung cancer tends to be younger and today's social life is under great pressure, and young and middle-aged patients have heavy work and family tasks, resulting in physical and mental exhaustion and lower physical activity levels [26]. Patients with perceived high disease severity had lower levels of physical activity. The reason is that a considerable number of patients believe that their condition is poor and increasing their activity will lead to relapse or aggravation of the disease, so they choose to sit still for recuperation [27].

Patients with high exercise self-efficacy were more physically active. On the contrary, patients with low exercise self-efficacy are more likely to suffer from insufficient physical activity, which is consistent with the findings of Qiu Pingping et al. [28]. Self-efficacy (Self-efficacy) refers to people's judgment on the organization and execution ability of the action process required to complete their own behavioral goals [29]. Sports self-efficacy is the embodiment of positive psychology applied to the field of sports. Many physical and mental problems are caused by the disease and treatment of lung cancer patients, as well as the influence of the traditional thinking of “more rest when sick” may lead to lung cancer patients being not fully aware of the benefits of exercise, or even knowing that exercise is beneficial, but due to the impact on their physical and mental conditions. Worry and lack of confidence in exercise ability, i.e., low exercise self-efficacy, both prevent lung cancer patients from benefiting from exercise. As a behavioral predictor, exercise self-efficacy is closely related to the exercise level and compliance of cancer patients, suggesting that the lack of exercise in lung cancer patients can be improved by improving the self-efficacy level of lung cancer patients [30].

Patients with a low perception of social support are more likely to suffer from insufficient physical activity, which is consistent with the findings of Yu Xiaomei et al. [27]. Social support is an important variable in promoting patient participation in physical activity. [31, 32]. Patients have close relationships with family members, and support and encouragement from family members, especially spouses, play a very important role.

The higher the patient's exercise self-efficacy and perceived social support scores, the higher the level of physical activity. Exercise self-efficacy is a good predictor of exercise behavior. Studies have shown [33] that exercise self-efficacy is related to individual exercise plan commitment and exercise persistence. Individuals with high exercise self-efficacy are more inclined to take the initiative to formulate and abide by exercise plans. Even if you encounter difficulties, you will try your best to overcome the obstacles and continue to exercise [34]. The more support a patient feels from relatives, friends, colleagues, and patients, the more secure the timing, intensity, and persistence of physical activity. It is recommended that medical staff start from enhancing the patient's sense of self-efficacy in sports and understanding of social support and taking relevant measures, such as explaining the benefits and safety of physical activity in detail, enhancing patients' exercise confidence, encouraging family members to participate in the patient's rehabilitation plan, and holding regular patient friendship meetings, and other activities to improve the physical activity level of lung cancer surgery patients.

## 5. Conclusions

The level of physical activity of patients undergoing lung cancer surgery needs to be further improved, and age, perceived disease severity, exercise self-efficacy, and perceived social support are the influencing factors. Physical activity levels were positively correlated with exercise self-efficacy and perceived social support. According to the age and characteristics of lung cancer surgery patients, medical staff can target young and middle-aged patients and patients who believe that they have a serious condition and enhance the sense of sports self-efficacy and social support for lung cancer surgery patients. This study also has certain limitations, such as studying patients from a single medical institution and having a limited sample size. In the future, multicenter and large-sample studies can be carried out to further explore the related factors of physical activity in patients with lung cancer surgery.

## Figures and Tables

**Figure 1:** Correlation scatter diagram of the physical activity level and sport self-efficacy.

**Figure 2:** Correlation scatter diagram of the physical activity level and understanding social support.

**Table 1:** Univariate analysis of physical activity levels in lung cancer surgery patients with different characteristics (*n* = 145).

Indexes	Number of cases	Physical activity level			*X* ^2^/*z* score	*P* score
		Insufficient/mildly deficient	Moderate	Active		
*Gender*					−0.358	0.721
Male	57	19(33.3%)	17(29.8%)	21(36.8%)		
Female	88	24(27.3%)	41(46.4%)	23(26.1%)		

*Body mass index*					0.657	0.720
20-25	73	21(28.8%)	29(39.7%)	23(31.5%)		
＜20	11	4(36.4%)	5(45.5%)	2(18.2%)		
＞25	61	18(29.5%)	24(39.3%)	19(31.1%)		

*Age*					7.606	**0.022**
＜40 year	11	7(63.6%)	3(27.3%)	1(9.1%)		
40-60 year	86	28(32.6%)	31(36.0%)	27(31.4%)		
＞60 year	48	8(16.7%)	24(50.0%)	16(33.3%)		

*Smoking*					−1.049	0.294
No	118	36(30.5%)	49(41.5%)	33(28.0%)		
Yes	27	7(25.9%)	9(33.3%)	11(40.7%)		

*Marriage*						
Yes	138	40(29.9%)	55(39.9%)	43(31.2%)	−1.021	0.307
No or others	7	3(42.9%)	3(42.9%)	1(14.3%)		

*Having children*					−1.646	0.100
No	11	5(45.5%)	5(45.5%)	1(9.1%)		
Yes	134	38(28.4%)	53(39.6%)	43(32.1%)		

*Education*					0.344	0.842
Graduate and above	12	3(25.0%)	5(41.7%)	4(33.3%)		
Undergraduate and college	51	18(35.3%)	13(25.5%)	20(39.2%)		
High school and below	82	22(26.8%)	40(48.8%)	20(24.4%)		

*Work status before hospitalization*					8.611	0.013
Full-time work	56	25(44.6%)	19(33.9%)	12(21.4%)		
Part-time work	18	5(27.8%)	5(27.8%)	8(44.4%)		
Does not work	71	13(18.3%)	34(47.9%)	24(33.8%)		

*Payment of medical expenses*					3.615	0.306
Self-pay	3	2(66.7%)	1(33.3%)	0(0.0%)		
Reimbursed	6	4(66.7%)	0(0.0%)	2(33.3%)		
Medical Insurance/Commercial Insurance	125	35(28.0%)	50(40.0%)	40(32.0%)		
New rural cooperative medical system	11	2(18.2%)	7(63.6%)	2(18.2%)		

*Per capita monthly household income*					3.473	0.324
¥ 0-2999	16	6(37.5%)	9(56.3%)	1(6.3%)		
¥ 3000-4999	63	16(25.4%)	28(44.4%)	19(30.2%)		
¥ 5000-9999	48	15(31.3%)	14(29.2%)	19(39.6%)		
≥ ¥ 10000	18	6(33.3%)	7(38.9%)	5(27.8%)		

*Economic Burden of Disease*					2.583	0.275
Light	20	5(25.0%)	6(30.0%)	9(45.0%)		
Moderate	103	32(31.1%)	45(43.7%)	26(25.2%)		
Heavy	22	6(27.2%)	7(31.8%)	9(40.9%)		

*Primary carrier*					0.211	0.900
Spouse	101	31(30.7%)	40(39.6%)	30(29.7%)		
Sons and daughters	32	8(25.0%)	14(43.8%)	10(31.3%)		
Others	12	4(33.3%)	4(33.3%)	4(33.3%)		

*Degree of understanding of the disease*					0.6673	0.716
Very understanding	33	11(33.3%)	11(33.3%)	11(33.3%)		
General understanding	102	30(29.4%)	43(42.2%)	29(28.4%)		
Poor understanding	10	2(20.0%)	4(40.0%)	4(40.0%)		

*Degree of understanding of disease prognosis*					5.187	0.075
Very understanding	27	7(25.9%)	8(29.6%)	12(44.4%)		
General understanding	100	32(32.0%)	45(45.0%)	23(23.0%)		
Poor understanding	18	4(22.2%)	5(27.8%)	9(50.0%)		

*Perceived severity of illness*					37.982	<0.001
Very serious	29	17(58.6%)	12(41.4%)	0(0.0%)		
Generally serious	85	24(28.2%)	39(45.9%)	22(25.9%)		
Not severe	31	2(6.5%)	7(22.6%)	22(71.0%)		

*Number of lesions*					−0.742	0.458
Single	91	24(26.4%)	39(42.9%)	28(30.8%)		
Multiple	54	19(35.2%)	19(35.2%)	16(29.6%)		

*Underlying disease*					−0.765	0.444
No	64	17(26.6%)	26(40.6%)	21(32.8%)		
Yes	81	26(32.1%)	32(39.5%)	23(28.4%)		

**Table 2:** Assignment table for unordered multiclass logistic regression analysis.

Factors	Variables	Assignment
Total exercise self-efficacy score	X1	Continuous variable
Comprehend social support total score	X2	Continuous variable
Age	X3	Continuous variable
Work status before hospitalization	X4	Works fine = 0, not working = 1
Perceived severity of illness	X5	Not serious = 0, very serious = 1

**Table 3:** Unordered multiclass logistic regression analysis of physical activity in patients with lung cancer surgery.

Indexes	Physically active			Physical inactivity/mild insufficiency		
	*p*	OR	95% CI	*P*	OR	95% CI
Total exercise self-efficacy score	<0.001	1.034	1.017∼1.052	<0.001	0.950	0.927∼0.974
Comprehend social support total score	0.760	1.009	0.953∼1.068	0.025	0.940	0.890∼0.992
*Age*	0.402	1.036	0.954∼1.126	0.023	0.916	0.850∼0.988

Work status before hospitalization						
Works fine	0.300	0.319	0.037∼2.768	0.805	0.776	0.103∼5.839
Not working	0.746	0.720	0.098∼5.288	0.436	0.437	0.064∼3.507

*Perceived severity of illness*						
Very serious		—	—	0.967	1.030	0.249∼4.271
Not severe	0.009	6.108	1.567∼23.803	0.798	0.727	0.063∼8.349

The independent variable work status before hospitalization and the perceived severity of the disease are taken as reference levels for taking part in work and general severity, respectively; the reference level of the dependent variable is moderate physical activity (patients who are not physically active in the perceived very severity of their disease, so no relevant value is discussed.).

**Table 4:** Physical activity level and sport self-efficacy, understanding social support in patients with lung cancer surgery Pearson correlation analysis (*n* = 145).

Indexes	Physical activity level	
	*R*	*P*
Sport self-efficacy	0.794	<0.001
Understanding social support	0.637	<0.001

## Data Availability

The data can be obtained from the author upon reasonable request.
